The article "Clinical Analysis of Echocardiography and Serum IL-6 and TNF-α Changes in Pregnant Women with Hypertension" was retracted in 2023. Reasons: signs of a paper mill; suspected computer-generated content; unreliable results or conclusions; lack of ethics approval or compliance.

# Clinical Analysis of Echocardiography and Serum IL-6 and TNF-*α* Changes in Pregnant Women with Hypertension

**DOI:** 10.1155/2022/9299746

**Published:** 2022-08-30

**Authors:** Ying Liu, Xiaolin Hou, Mei Yu, Jin Zhou

**Affiliations:** ^1^Obstetrical Department VIII, The Fourth Hospital of Shijiazhuang (The Obstetrics and Gynecology Hospital of Hebei Medical University), Shijiazhuang, Hebei 050000, China; ^2^Prenatal Diagnosis Center, The Fourth Hospital of Shijiazhuang (The Obstetrics and Gynecology Hospital of Hebei Medical University), Shijiazhuang, Hebei 050000, China; ^3^Health Care Center, The First Hospital of Hebei Medical University, Shijiazhuang, Hebei 050000, China

## Abstract

In order to explore the changes and clinical significance of serum TNF-*α* and IL-6 and ET levels in the pathogenesis of hypertensive disorders of pregnancy (HDIP), echocardiography, and serum IL-6 and TNF-*α* changes in pregnant women with a hypertensive disorder, a clinical analysis method was proposed. A retrospective analysis of 59 pregnant women who visited the obstetrics department of a provincial hospital was divided into 2 groups. The normal control group consisted of 32 normal, uncomplicated pregnant women; the preeclampsia group included 27 patients with systolic blood pressure > 140 mmHg and/or diastolic blood pressure > 90 mmHg who developed proteinuria after 20 weeks of gestation. The levels of TNF-*α* and IL-6 in serum of normal pregnant women and pregnant women with preeclampsia were detected by enzyme-linked immunosorbent assay (ELISA). The results showed that compared with normal pregnant women, the serum levels of TNF-*α* and IL-6 in the early pregnant women of Zizhi were significantly increased, and the trend of increased TNF-*α* and IL-6 levels was related to the severity of complications. With the mean pulmonary arterypressure > 50 mmHg, the serum TNF-*α* level of pregnant women was significantly higher than that of pregnant women with mean pulmonary arterypressure < 50 mmHg. The analysis found that the serum levels of TNF-*α* and IL-6 in patients with hypoxic gestational hypertension were significantly increased, and the results of lung tissue immunohistochemistry also showed that serum TNF-*α* and IL-6 levels in patients with hypoxic gestational hypertension were significantly increased. And serum TNF-*α* and IL-6 levels were positively correlated with right ventricular systolic blood pressure (RVSP). *Conclusion*. This study revealed that the elevated levels of serum TNF-*α* and IL-6 are closely related to the pathophysiological process of gestational hypertension. Serum levels of TNF-*α* and IL-6 and ET were significantly increased, and the changes of serum TNF-*α* and IL-6 and ET levels had important clinical value for closely monitoring the severity of the disease and the development of the disease.

The article "Clinical Analysis of Echocardiography and Serum IL-6 and TNF-α Changes in Pregnant Women with Hypertension" was retracted in 2023. Reasons: signs of a paper mill; suspected computer-generated content; unreliable results or conclusions; lack of ethics approval or compliance.

## 1. Introduction

Pregnancy is a special physiological period for women, and various physiological indicators of the body will change, in order to facilitate the growth of the fetus in the mother and the later delivery. During pregnancy, the levels of progesterone and estrogen in pregnant women change significantly, and their serum levels reach their peaks in the third trimester; these hormones affect the synthesis, metabolism, and secretion functions of the liver and kidney. Pregnancy hypertension is a group of diseases associated with gestational hypertension, preeclampsia, and eclampsia; chronic hypertension is associated with complications of preeclampsia; pregnancy with complications of hypertension will increase with gestational age. Damage to pregnant women is shown in Figure 1; the effect can be reversible [1]. Hypertensive disease during pregnancy has always been a disease of great concern to obstetric workers, and it is a major risk factor for maternal and perinatal life and death. The incidence rate in China is 9.4%, and the reported incidence rate in foreign countries is 7%-12%, and the death caused by it accounts for 12% of maternal deaths; it is one of the main reasons that threatens the safety of mothers and babies and causes maternal death. In recent years, although researches on hypertensive disorders of pregnancy have emerged in an endless stream, so far, the pathogenesis of the disease has not been elucidated [2]. The main clinical manifestations of gestational hypertension are high blood pressure, heart and kidney failure, edema, proteinuria, convulsions, etc.; with the gradual development of the disease, some patients may have serious complications such as renal failure, premature birth, coma, and even death; among these complications, acute kidney injury (AKI) is the main complication and the leading cause of maternal miscarriage, preterm birth, fetal growth retardation, and maternal death [3]. Because the damage of renal function can be reversed in time through treatment in the early stage, and the renal function can be restored to normal, so early diagnosis and early treatment are recommended in clinical treatment.

## 2. Literature Review

Gabbay-Benziv et al. cultured trophoblast cells in vitro and detected inhibin A, indicating that there is mRNA encoding inhibin A in trophoblast cells [4]. Contro et al. showed that the expression of inhibin A was different in the trophoblast cells of normal pregnant women and women with preeclampsia, and the latter was higher than the former [5]. The results of a case-control study by Wang et al. showed that inhibin A was 295pg/L, with a sensitivity of 85.7%, a specificity of 98.5%, and an accuracy of 0.954, suggesting that inhibin A can be used as an indicator factor for early prediction of preeclampsia [6]. Fisher found that in women who developed hypertensive disorders of pregnancy in the second trimester, serum inhibin A levels were not different from those of normal pregnant women [7]. Yi et al. suggested that the serum inhibin A concentration of pregnant women in the second trimester was not associated with the occurrence of preeclampsia [8]. Kumar et al. showed that activin A can be used as an independent risk factor for predicting early-onset preeclampsia, and it is associated with cell-free fetal DNA, both of which are higher in the serum of pregnant women with preeclampsia [9]. Roukoz compared 50 cases of preeclampsia and 250 normal cases at 11-13 weeks of gestation and 30-33 weeks of gestation. It was found that there was no significant difference in serum activin A levels between the two groups at 11-13 weeks of gestation, but it was significant at 30-33 weeks of gestation, and combined with serum activin A levels at 30-33 weeks of gestation and the general clinical data of pregnant women, it was possible to detect 50% of patients with preeclampsia [10]. Combined with PP13, PAPP-A, ADAM12, activin A, inhibin A, and uterine artery Doppler hemodynamics in the second trimester, the sensitivity for predicting preeclampsia can reach 60%-80%, and the specificity can reach 60%-80%; when the specificity of activin A combined with PI value in predicting preeclampsia was 90%, the sensitivity was only 57%. Iwahasi et al. took the serum of pregnant women with early-onset preeclampsia and normal pregnant women and detected PAPP-A in serum; using median comparison, they found that pregnant women with early-onset preeclampsia were lower than normal pregnant women (0.80 MoMs vs. 1.05 MoMs, *P* = 0.005), combined with RBP4, predicting a 34% increase in DR in early-onset preeclampsia, and PAPP-A can be used as a useful indicator for predicting early-onset and severe preeclampsia [11].

The article "Clinical Analysis of Echocardiography and Serum IL-6 and TNF-α Changes in Pregnant Women with Hypertension" was retracted in 2023. Reasons: signs of a paper mill; suspected computer-generated content; unreliable results or conclusions; lack of ethics approval or compliance.

## 3. Research Methods

### 3.1. Echocardiographic Assessment of Pain in Gestational Hypertension

Echocardiography was performed by an echocardiographer with more than 10 years of clinical experience. The following points should be noted during the examination: the echocardiographic image grade should not be lower than grade C. The calculated value of pulmonary artery pressure is uniformly plus 5 mmHg (mild) on the basis of the tricuspid transvalvular pressure difference. The report should include tricuspid regurgitation velocity, transvalvular pressure gradient, and estimated pulmonary systolic pressure. If the pulmonary artery pressure is above 50 mmHg, it should be regarded as pathological and should not be treated as a normal pregnant woman.

The main evaluation indicators included the following echocardiographic indicators:

1. Longitudinal axis of left ventricle: aortic main diameter, left atrium diameter, interventricular septum thickness, left ventricular end diastolic diameter, left ventricular systolic end diameter, and left ventricular posterior wall thickness
2. Long-axis view of the pulmonary trunk: pulmonary trunk
3. Right heart measurements (apical four-chamber view): right ventricular base diameter, right atrium diameter, left ventricular mass index (LVMI), and tricuspid annular presystolic amplitude (TAPSE)
4. Measurement of left ventricular systolic function: left ventricular ejection fraction (EF), left ventricular short-term shortening (FS), stroke rate (SV), and minute output (cardiac output, CO)
5. Measurement of left ventricular diastolic function: spectral diagram of mitral valve blood flow: E peak, A peak, E/A, and E peak time delay (EDT); Doppler imaging TDI: early systolic peak velocity (S), early diastolic peak velocity (e′), and late diastolic peak velocity (a′)
6. Pulmonary arterial pressure measurement: tricuspid regurgitation velocity, tricuspid transvalvular pressure gradient, and estimated pulmonary artery systolic pressure

At the same time, this study also recorded the subjects' age, heart rate, height, and weight and asked the patients their prepregnancy weight as their standard weight [12].

The inside diameter of the left ventricle and its walls are measured against the longitudinal axis of the left ventricle. When measuring, select an area perpendicular to the longitudinal axis and measure at or near the apex of the mitral valve. An electrical cursor is placed at the junction of the myocardial wall and the heart chamber, between the ventricular wall and the pericardium. The inner diameter of the chamber can be obtained with 2D ultrasound guided M-mode, but a better method is to obtain it directly with 2D ultrasound images, which avoids the bevel of the ventricle and makes it more accurate.

Fractional shortening can be obtained from a 2D guided M-mode image, but it is best to measure radial lines directly on the 2D image. In the case of segmental wall motion abnormalities caused by coronary heart disease or conduction abnormalities, the overall function of the left ventricle based on diameter measurements is very problematic. In patients with uncomplicated hypertension, obesity, or valvular disease, such as without clinically confirmed myocardial infarction, such segmental differences are rare, so fractional shortening can provide clinically useful information. In patients with basal LV but increased medial and left venous volume, the LV value was higher than that of the basal LV.

The article "Clinical Analysis of Echocardiography and Serum IL-6 and TNF-α Changes in Pregnant Women with Hypertension" was retracted in 2023. Reasons: signs of a paper mill; suspected computer-generated content; unreliable results or conclusions; lack of ethics approval or compliance.

Calculate the fraction (EF) that differs from the mean values of the left ventricular systolic volume (EDV) and the left ventricular diastolic volume (ESV), and its formula is as follows:

(1) $$\begin{array}{c} EF=\frac{\left(EDV-ESV\right)}{EDV}. \end{array}$$

Left heart measurement should be done in 2D or 3D. The interface between the thick myocardium and the left ventricular cavity is closed, and the entire contour is closed with a straight line to the mitral annulus. Longer lines were selected in apical two-chamber view and four-chamber view. Left ventricular volume should be measured at apical four-chamber and two-chamber views. Select the largest left ventricular area of the left ventricle, and try not to shorten the left ventricle and underestimation of the left ventricular volume [13]. When examining, reduce the depth of the image to focus on the left ventricular cavity, which reduces the chance of left ventricular shortening; it also minimizes errors in tracing the endocardium.

In the left heart, M type, 2D, and 3D are valid methods for counting left heart. All measurements should be made at the end of the diastole (the frame before the mitral valve closes, or the frame with the largest central chamber diameter or volume during the cardiac cycle). Left ventricular diastolic diameter and wall thickness measured with M type or 2D both rely on geometric models to calculate the left ventricular diameter, while 3D ultrasound can measure LV volume directly, all the way to change the volume to size by taking the volume of myocardial by myocardial density. At the same time, the study also recorded age, heart rate, height, and weight and asked patients their weight before pregnancy based on their weight.

### 3.2. Correlation between Serum Markers TNF-a and IL-6 Levels and Gestational Hypertension

#### 3.2.1. Study Population

The subjects of the analysis were the records of pregnant women who delivered inpatients in the obstetrics department of a provincial hospital between May 2021 and May 2022. The study included 59 participants who were divided into two groups. One of the groups was 27 pregnant women who suffered from prepain and gave birth in our hospital and was designated as the prepain group. Significant symptoms are two or more wet measurements of pregnant woman blood pressure after 20 weeks of gestation, systolic blood pressure > 140 mmHg, and/or diastolic pressure > 90 mmHg, and the measurement time was at least 4 hours, proteinuria. In another group, 32 pregnant women who gave birth without problems during pregnancy were identified as the normal control group. The gestational age and maternal age of pregnant women in pre-Ziton and control groups were always similar. All pregnant women had one pregnancy, and this study did not include women with high blood pressure, heart disease, kidney disease, or type 1 or type 2 diabetes.

The article "Clinical Analysis of Echocardiography and Serum IL-6 and TNF-α Changes in Pregnant Women with Hypertension" was retracted in 2023. Reasons: signs of a paper mill; suspected computer-generated content; unreliable results or conclusions; lack of ethics approval or compliance.

#### 3.2.2. Methods

The analysis groups were set up as follows: (1) normoxia control pregnancy group, (2) pregnancy-induced hypertension group, and (3) treprostinil treatment group [14]. Blood samples for TNF-*α* and IL-6 were collected from the heart and stored at -80°C.

*(1) Right Ventricular Systolic Blood Pressure Detection*. Pentohexidine was administered intravenously (30 mg/kg) was injected intravenously, and the trachea was intubated and placed in a well-ventilated environment. The thoracic cavity was opened, a PE-50 polyethylene tube was inserted into the right ventricle, and the right ventricular systolic pressure was collected by energy-Lab data collection.

*(2) Extraction of Total RNA*. Use TRIzol to extract total RNA from lung tissue, and the specific operation steps are as follows:

- 50 mg of lung tissue was added to 1 ml of TRIzol, placed in liquid nitrogen, and homogenized by a homogenizer
- The homogenized samples were placed at room temperature for 5 min to completely separate nucleic acid and protein
- Add 200 *μ*l chloroform, shake for 15 s, and allow to stand at room temperature for 1 min
- Centrifuge at 10,000 × *g* for 15 min at 4° C. After centrifugation, the sample was divided into three layers: the lower layer (red organic phenol-chloroform phase), the middle layer, and the upper colorless aqueous phase. RNA in the upper colorless aqueous phase
- Transfer the colorless water-free phase to a new EP tube, add 500 isopropanol, and allow to stand at room temperature for 10 minutes
- Centrifuge at 10,000 × *g* for 15 min at 4° C to remove the top layer
- To wash the RNA pellets, add 1 ml of precooled 75% ethyl alcohol, centrifuge at 7500 × *g* at 40° C for 5 min, and remove the top layer
- Dry the RNA pellets at room temperature, adding about 50 (depending on the size of the pellets) RNase-free water, and store at 80° C to dissolve the RNA pellets

*(3) Reverse Transcription of RNA*. cDNA was synthesized in vitro by Moloney's leukemia virus reverse transcriptase (M-MLV RT), and the operation steps were as follows:

- Add the following components in Table 1 to a nuclease-free microcentrifuge tube

(b) After the mixture was heated at 70°C for 5 minutes, it was quickly cooled on ice for 5 minutes
(c) After a brief centrifugation, the following components were added as shown in Table 2

(d) The components were mixed gently and reacted at room temperature for 10 minutes and then heated at 45°C for 50 minutes
(e) Heat at 70°C for 15 minutes to stop the reaction

*(4) Real-Time Quantitative PCR (Real-Time Quantitative PCR)*. The SYBR∗ Pemix Ex Tag™ kit was used for the real-time fluorescent quantitative PCR reaction. The specific steps are as follows:

- Prepare the reaction system according to the components in Table 3 (the preparation should be carried out on ice)

(b) Run the RT-PCR reaction. The reaction process is shown in Table 4

*(5) Immunohistochemistry*.

- Dewaxing

- Paraffin sections of 4 thickness were sequentially placed in 100% xylene (a) and 100% xylene (b) at 37°C for 15 min each
- The slices were sequentially placed in 100% ethanol-100% ethanol-95% ethanol-80% ethanol-70% ethanol-plus % ethanol for 2 minutes each
- The slices were soaked in double-distilled water for 2 minutes and repeated 3 times [15]

(ii) Antigen Retrieval

- After dewaxing, the samples were placed in 3% H_2_O, treated at room temperature for 15 minutes, and then soaked in double-distilled water for 2 minutes, repeating 3 times
- Preheat the 0.1 m citric acid solution in the microwave for 3 minutes, quickly put the slices into the sodium citrate solution, and continue to boil for 15 to 20 minutes

(iii) Serum Blocking

- The samples were cooled for 30 minutes and then soaked in double-distilled water for 2 minutes, repeating 3 times
- After the double-distilled water on the tissue evaporated, immediately add serum-containing peroxidase blocking agent to block, and incubate at 37°C for 30 minutes

(iv) Antibody Incubation

- Incubate with primary antibody, incubate at 37°C for 30 minutes, discard the blocking solution, add TNF-*α* or IL-6 antibody, and incubate at 4°C overnight
- After incubation with the secondary antibody, after recovering the primary antibody, the samples were washed three times with PBS for 5 minutes each time. After washing, biotinylated rabbit anti-goat secondary antibody was added and incubated at room temperature for 15 minutes

(v) Color Rendering

After adding the chromogenic substrate 3,3-diaminobenzidine (3,3-diaminobenzidine DAB), the sample reacts with horseradish peroxidase-labeled streptavidin, and the color is observed under a microscope. Rinse with clean water after sufficient color development.

(vi) Counterstaining

The slides were washed in double-distilled water for 3 minutes and then counterstained with hematoxylin for 30 seconds after repeated 3 times. Rinse twice with tap water for 6 minutes each time.

(vii) Dehydration

The slides were washed in double-distilled water for 3 minutes, repeated 3 times and then placed in 70% ethanol-80% ethanol-90% ethanol-95% ethanol-100% ethanol-100% ethanol-xylene-xylene for 2 minutes, and finally soaked in xylene [16].

(viii) Cover Sheet

Drop the neutral gum next to the tissue, cover with a coverslip, and lay down one side first and then the other to avoid air bubbles. Dry the sealed slides in a 65°C oven overnight.

The article "Clinical Analysis of Echocardiography and Serum IL-6 and TNF-α Changes in Pregnant Women with Hypertension" was retracted in 2023. Reasons: signs of a paper mill; suspected computer-generated content; unreliable results or conclusions; lack of ethics approval or compliance.

#### 3.2.3. Data Analysis

Unless otherwise specified, all data are indicated as average ± SD. Tukey's post hoc tests were performed using Prism version 5 software to determine whether there was a discrepancy between the control panel and the test group using *t*-test or unilateral ANOVA. The correlation of the differences was evaluated by Pearson's correlation coefficient [17]. *P* < 0.5 was considered statistically significant.

## 4. Analysis of Results

### 4.1. Clinical Characteristics of Participants

The clinical characteristics of all participants in the concept of pregnancy are shown in Table 5. There were no significant differences in marital, birth history, ethnicity, or education level of control group and antenatal hypertension group [18]. However, in pregnant women in the gestational hypertension group with the same gestational and maternal age, compared with the control group, their prepregnancy body mass index was higher, and they had a higher incidence of anemia.

### 4.2. The Serum Levels of TNF-*α* and IL-6 Increased in the Serum of Pregnant Women in the Early Stage of Zitong

Blood levels of TNF-*α* and IL-6 were detected by ELISA assay, and blood levels of TNF-*α* in pregnant women were detected at an earlier stage than in the control group. The Ziji group has grown. In addition, we found plasma levels of TNF-*α* and IL-6 in the blood, due to which pregnancy causes patients with pulmonary arterial hypertension, and pathophysiological changes in pulmonary arterial hypertension increase morbidity and mortality for pregnant women. Hypertension during pregnancy is determined by the average value of pulmonary arterial pressure [19]. We retrospectively analyzed the hemodynamic data of 27 pregnant women with preeclampsia and serum TNF-*α* levels of pregnant women with mean pulmonary arterypressure ≥ 50 mmHg, significantly higher than the average pulmonary arterypressure < 50 mmHgin pregnant women (Figure 2).

Plasma TNF-*α* levels in pregnant women mean pulmonary arterial pressure ≥ 50 mmHg is higher than in pregnant women who mean pulmonary arterial pressure less than 50 mmHg. In the meandata + standarddeviation,*P* < 0.01means the significant difference compared to the control group. Levels of IL-6 in pregnant women, which means pulmonary arterial pressure ≥ 50 mmHg and pulmonary arterial pressure less than 50 mmHg, meet TNF-*α* levels. Based on the above results, serum levels of TNF-*α* and IL-6 were significantly elevated in pregnant women with gestational hypertension and were associated with the severity of complications.

The article "Clinical Analysis of Echocardiography and Serum IL-6 and TNF-α Changes in Pregnant Women with Hypertension" was retracted in 2023. Reasons: signs of a paper mill; suspected computer-generated content; unreliable results or conclusions; lack of ethics approval or compliance.

### 4.3. Drug Therapy Can Reduce Serum TNF-*α* and IL-6 Levels in Hypoxia-Induced Gestational Hypertension

To determine which plasma TNF-*α* and IL-6 levels can be used as biomarkers in prenatal hypertension, we examined blood TNF-*α* and IL-6 levels in pregnancy samples treated with treprostinil [20]. Treprostinil is a group of vasodilators used to treat pulmonary arterial hypertension. Three recent studies have shown that treprostinil is effective in treating pulmonary hypertension in pregnant women with hypoxia-induced hypertension. Compared with normoxic administration, the right ventricular systolic blood pressure was increased during hypoxia, and treprostinil treatment reduced the right ventricular systolic blood pressure during hypoxia-induced gestational hypertension. Treprostinil treatment has been shown to significantly reduce the incidence of gestational hypertension due to hypoxia.

## 5. Conclusion

Studies have shown that blood TNF-*α* and IL-6 levels are higher in pregnant women with higher blood pressure than in pregnant women, indicating that TNF-*α* and IL-6 levels are higher, associated with high blood pressure. Right ventricular systolic blood pressure was significantly higher in patients exposed to hypoxia than in normoxic controls. When treated with treprostinil, right ventricular systolic blood pressure in hypoxic-induced hypertensive depression of pregnancy was decreased. Plasma levels of TNF-*α* and IL-6 can also be used in the treatment and prevention of gestational hypertension.

## Figures and Tables

**Figure 1:** Effects of gestational hypertension.

**Figure 2:** Relationship between mean pulmonary arterial pressure and serum TNF-*α* level in pregnant women with gestational hypertension.

**Table 1:** Nuclease-free microcentrifuge tube components.

Reagent	Volume
Random primer	150 ng
Total RNA	500 ng
Nuclease-free water replenishes the total volume	14 *μ*l

**Table 2:** Components added after brief centrifugation.

Reagent	Volume
M-MLV RT 5 × reaction buffer	5 *μ*l
dATP, 10 mM	1.25 *μ*l
dCTP, 10 mM	1.25 *μ*l
dGTT, 10 mM	1.25 *μ*l
dTTP, 10 mM	1.25 *μ*l
M-MLV RT (H-) point mutant	1 *μ*l (50–100 units)
Nuclease-free water replenishes the total volume	25 *μ*l

**Table 3:** Components of the distribution reaction system.

Reagent	Volume
SYBR∗ Premix Ex Tag™ (2×)	12.5 *μ*l
PCR forward primer (10 *μ*M)	1 *μ*l
PCR reverse primer (10 *μ*M)	1 *μ*l
DNA template	2 *μ*l
ddH_2_O	8.5 *μ*l
Total	25 *μ*l

The article "Clinical Analysis of Echocardiography and Serum IL-6 and TNF-α Changes in Pregnant Women with Hypertension" was retracted in 2023. Reasons: signs of a paper mill; suspected computer-generated content; unreliable results or conclusions; lack of ethics approval or compliance.

**Table 4:** RT-PCR reaction process.

Cycle	Temperature	Duration
Loop 1 (2×)	95°C	10s
Loop 2 (40×)	95°C	10s
	60°C	30s
Cycle 3 (dissolution curve)	90 °C	10s
	60°C	1 min
	95°C	10s

**Table 5:** Summary of clinical information of 59 pregnant women.

Basic features	Gestational hypertension group (*n* = 27)	Control group (*n* = 32)
Mean age of mother (years)	27.3	28.2
Prepregnancy body mass index BMI (kg/m^2^)	25.2	17.8
Anemia	9/27 (33.3%)	1/32 (3.1%)
Asian ethnic group	27/27 (100.0%)	32/32 (100.0%)
Reproductive history		
History of spontaneous abortion (>3)	3/27 (11.1%)	4/32 (12.5%)
Number of pregnancies (>3)	7/27 (25.9%)	9/32 (28.1%)

## Data Availability

The data used to support the findings of this study are available from the corresponding author upon request.
